# PknE, a Serine/Threonine Protein Kinase of *Mycobacterium tuberculosis* Initiates Survival Crosstalk That Also Impacts HIV Coinfection

**DOI:** 10.1371/journal.pone.0083541

**Published:** 2014-01-08

**Authors:** Dinesh Kumar Parandhaman, Luke Elizabeth Hanna, Sujatha Narayanan

**Affiliations:** 1 Department of Immunology, National Institute for Research in Tuberculosis, Chennai, TamilNadu, India; 2 Department of Clinic Research, HIV division, National Institute for Research in Tuberculosis, Chennai, TamilNadu, India; University of Maryland, United States of America

## Abstract

Serine threonine protein kinases (STPK) play a major role in the pathogenesis of *Mycobacterium tuberculosis*. Here, we examined the role of STPK *pknE*, using a deletion mutant Δ*pknE* in the modulation of intracellular signaling events that favor *M. tuberculosis* survival. Phosphorylation kinetics of MAPK (p38MAPK, Erk½ and SAPK/JNK) was defective in Δ*pknE* compared to wild-type infected macrophages. This defective signaling dramatically delayed and reduced the phosphorylation kinetics of transcription factors ATF-2 and c-JUN in Δ*pknE* infected macrophages. MAPK inhibitors instead of reducing the phosphorylation in Δ*pknE* infected macrophages, revealed crosstalks with Erk½ signaling influenced by SAPK/JNK and p38 pathways independently. Modulations in intra cellular signaling altered the expression of coreceptors CCR5 and CXCR4 in Δ*pknE* infected macrophages. In conclusion, *pknE* plays a role in MAPK crosstalks that enables intracellular survival of *M. tuberculosis*. This survival strategy also impacts HIV/TB coinfection.

## Introduction

The global incidence of tuberculosis (TB) caused by *Mycobacterium tuberculosis* (MTB) has increased due to the emergence of drug resistant strains and HIV coinfection [1]. The adaptation of MTB in hostile environments is regulated by serine/threonine protein kinases (STPK). Among the 11 STPKs encoded by MTB, *pknE*, *pknG*, *pknH*, *pknI* and *pknK* play a role in its intracellular survival [2]–[6].

STPKs are prime targets for new drug discovery and share only 30% homology with their human counterparts [7]. The likelihood of STPKs in mediating intracellular signaling events in the host remains elusive. However, two other MTB genes, *eis* and *mPTPB* were reported to play a role in the modulation of host intracellular signaling [8], [9].

Mitogen activated protein kinase (MAPK) cascades are evolutionarily conserved signaling pathways in eukaryotes that play a role in cell proliferation, cell differentiation, cell movement and cell death [10]. MAPK family is divided into four main subfamilies namely extracellular regulated kinases 1 and 2 (Erk½), Jun N-terminal kinases (JNKs), p38 MAPK and Erk5 [11]. MAPKs were reported to have cooperated signaling with shared substrates [12]. Erk½ pathway activated by growth factors and mitogens plays a major role in regulating cell proliferation and differentiation. On the other hand, environmental stress, inflammatory cytokines and stress-dependent apoptosis stimulate p38 and SAPK/JNK pathways [10]. Activated MAPKs signal the transcription factors to regulate the expression of cytokines and iNOS [10]. Studies on *Mycobacterium* have shown the suppression of MAPK signaling as a mechanism to prevent macrophage activation [10].

TB predominates in HIV-infected individuals due to weakened immune functions that lead to reactivation of latent MTB. Disease progression in HIV/TB coinfected individuals is accelerated by both MTB and HIV [13]. Cellular components of MTB are known to regulate coreceptors CXCR4 and CCR5 involved in HIV entry [14], but the molecular mechanisms underlying this phenomenon are not well-understood. Previously, we reported that *pknE* expressed under nitric oxide (NO) stress suppresses multiple apoptotic pathways thereby supporting intracellular survival of MTB and that purified PknE cross-reacts with SAPK/JNK antibody [3].

In the present study, the influence of *pknE* on intracellular signaling that favors MTB survival and its impact on the outcome of HIV/TB coinfection were studied. Our data shows that *pknE* of MTB influences the crosstalk between the MAPK pathways to regulate inflammation and HIV/TB coinfection.

## Methods

### Bacterial strains and culture conditions

MTB H_37_Rv (Rv, wild-type), H_37_Rv*pknE*::hyg (Δ*pknE*, *pknE* deletion mutant) and complemented H_37_Rv*pknE* strain (CΔE) were grown in Middlebrook 7H9 broth as reported earlier with 50 µg/ml of hygromycin and 20 µg/ml of kanamycin when required [3].

### Cell culture, infection, inhibitors and nitrate stress experiments

THP-1 cells were maintained, differentiated and infected as reported earlier [15]. Cells were pretreated for 1 h with inhibitors of Akt (Wortmannin, 100 nM), arginase (N^ω^-Hydroxy-nor-L-arginine diacetate, 100 µM), caspase-8 (Z-IETD-FMK, 25 µmol/L), caspase-9 (Z-LEHD-FMK, 25 µmol/L), Erk½ (PD98059, 20 µM), p38 (SB203580, 10 µM), SAPK/JNK (SP600125, 10 µM) and TP53 (pifithrin-α, 5 µmol/L) purchased from Calbiochem, USA, and infected with MTB strains. For nitrate stress experiments, post-infection with MTB, the cells were treated with 10 mM sodium nitroprusside (SNP) as reported earlier [15].

### Western blotting

Cell lysates were prepared as reported earlier [15] and the immunoblots were probed with rabbit anti-human polyclonal antibodies (Cell Signaling Technologies) against phospho and non-phospho Akt, p38, Erk½ and SAPK/JNK (1∶1000) and detected using horseradish peroxidase-conjugated goat anti-rabbit antibody (1∶300) (Amersham Biosciences).

### Transcription factor ELISA

Nuclear factors were isolated using the procedure reported earlier [16]. Briefly, 1×10^6^ THP-1 macrophages were lysed using 300 µl of buffer A (10 mM HEPES–KOH, pH 7.9, 1.5 mM MgCl_2_, 10 mM KCl, 0.5 mM DTT, 0.2 mM PMSF), centrifuged for 10 s at 15,000 g and the supernatants were labeled as cytosolic fraction. The cell pellet was resuspended in 200 µl of icecold buffer B (20 mM HEPES–KOH, pH 7.9, 25% glycerol, 420 nM NaCl, 1.5 mM MgCl_2_, 0.2 mM EDTA, 0.5 mM DTT, 0.2 mM PMSF), centrifuged at 15,000 g for 10 s and the supernatants were stored at −80°C until use. The concentration of proteins was quantified using bicinchoninic acid method (Sigma).

Trans-AM ATF-2, c-JUN and NF-kB kit from Active Motif (Carlsbad, CA) were used to determine the levels of ATF-2, c-JUN and p65NF-kB in nuclear extract. 2 µg of nuclear extract was added to wells coated with oligonucleotides containing the consensus binding site for the respective nuclear factors, followed by addition of primary antibody, horseradish peroxidase-conjugated secondary antibody and the substrate. The absorbance was read at 450 nm (with a reference wavelength at 650 nm). The specificity of the assay was monitored using competitive binding of wild-type or mutated consensus oligonucleotides before the addition of nuclear extracts.

### HIV/TB coinfection

24 h post-infection with MTB, THP-1 cells were infected with 500TCID_50_ of CCR5 (92UG005) and CXCR4 (92UG024)-tropic HIV-1 virus for 2 h at 37°C. Post infection extracellular virus was removed by wash using serum-free RPMI and replenished with RPMI containing 10% FBS. The supernatant was harvested on day 4 to estimate the viral p24 levels by sandwich ELISA (Perkin Elmer). Similarly, monocyte derived macrophages (MDM) were isolated from the blood received from healthy volunteers (Jeevan blood bank, http://www.jeevan.org/blood/index.html) after written informed consent approved by institutional ethics committee review board (NIRT IEC protocol number 2006 006) and the coinfection experiment was carried out as described above.

### Statistics

Statistical analysis was carried out using graph pad prism v5.0. One way and Two way ANOVA were used depending on the data and p value<0.05 was considered statistically significant.

## Results

### Δ*pknE* decreases phosphorylation of MAPKs

The phosphorylation kinetics of Erk½, p38MAPK and SAPK/JNK were compared in THP-1-derived macrophages infected with MTB strains Rv, Δ*pknE* and CΔE (complemented Δ*pknE*). Control cells and Lipopolysaccharide (LPS) were used as appropriate controls.

Rv-infected macrophages had increased levels of phosphorylation of Erk½, p38MAPK and SAPK/JNK from 30 min post-infection compared to controls (Figures 1A–C). In contrast, Δ*pknE*-infected macrophages abrogated the phosphorylation of Erk½ at 240 min (p<0.0001, for all the time periods), reduced the phosphorylation of p38MAPK at 60 min (p<0.0001) and selectively inhibited the phosphorylation of p46 subunit of SAPK/JNK at 120 min (p<0.0001) post infection compared to Rv-infected macrophages (Figures 1A–C). These data reveal that *pknE* modulates the MAPK signaling thereby providing a survival niche for MTB.

**Figure 1:** Δ*pknE* infected macrophages are defective in MAPK signaling. Controls (Ctrl, LPS) and infected cells were lysed post infection at varied time points and subjected to western blotting. The blots were probed with phospho A) Erk1/2, E) p38, and I) SAPK/JNK and their respective non phospho (C, G and I) antibodies. The results are from three independent experiments. Figures B, D, F, H, J, K, and L depict the corresponding densitometry values of phospho and nonphospho antibody probed blots. *, *** denotes p<0.05 and p<0.0001, when Δ*pknE* infected macrophages compared with Rv (one – way ANOVA). The abbreviations ctrl denotes control and LPS denotes lipopolysaccharide.

### Δ*pknE* decreases phosphorylation of ATF-2 and c-JUN while NF-kB is unaltered

Decreased MAPK signaling in Δ*pknE*-infected macrophages prompted us to study the expression of transcription factors ATF-2, c-JUN and NF-kB, the final targets for cellular activation.

Phosphorylation of ATF-2 and c-JUN in Rv-infected macrophages peaked at 60 min and returned to baseline at 240 min post-infection, while in Δ*pknE*-infected macrophages it peaked at 120 min and reached baseline levels at 240 min post-infection. Phosphorylation of ATF-2 and c-JUN in LPS-treated macrophages peaked at 120 min post-treatment and reached baseline values at 240 min post-infection (Figures 2A,2B). Phosphorylation kinetics of NF-kB was similar in both Rv and Δ*pknE*-infected macrophages (Figure 2C). CΔE was able to reverse the altered phosphorylation events observed in Δ*pknE*-infected macrophages.

**Figure 2:** Δ*pknE* infected macrophages have reduced expression of transcription factors. Nuclear fractions isolated post infection was subjected to DNA binding ELISA for A) ATF-2, B) c-JUN, and C) NF-kB. The results from three independent experiments are shown. The O.D values denote standard error of the means. *denote p<0.05 (Two way ANOVA) when Δ*pknE* versus Rv infected macrophages were compared.

This clearly shows that deletion of *pknE* reduces cellular inflammation due to delayed and reduced activation of transcription factors and reconfirms our previous finding that *pknE* contributes to inflammatory responses [15].

### MAPK signaling in Δ*pknE*-infected macrophages is unaltered in the presence of pathway-specific inhibitors

The inhibition of MAPK signaling by Δ*pknE*-infected macrophages was assessed using pathway-specific inhibitors. Surprisingly, p38MAPK, Erk½, SAPK/JNK or Akt inhibitors were unable to suppress the phosphorylation in Δ*pknE*-infected macrophages as observed in macrophages infected with Rv (data not shown).

### Δ*pknE* induces crosstalk between Erk½ and SAPK/JNK signaling

The absence of inhibition in the presence of MAPK and Akt inhibitors observed in Δ*pknE*-infected macrophages suggests two plausible facts; either Δ*pknE* induces phosphatases of MAPK differentially or that it initiates a crosstalk response. We chose to analyze Erk½ crosstalk based on its reduced expression in Δ*pknE*-infected macrophages and its role in cellular survival.

We performed crosstalk analysis between the Erk½ and SAPK/JNK pathways as reported in a previous study [17]. While Erk½ inhibitor did not affect SAPK/JNK phosphorylation, SAPK/JNK inhibitor reduced phosphorylation of Erk½ in Δ*pknE*-infected macrophages as compared to Rv-infected macrophages (Figure 3A). p38MAPK inhibitor also modestly reduced Erk½ phosphorylation in Δ*pknE*-infected macrophages when compared to Rv-infected macrophages (Figure 3B). Thus MTB is able to initiate crosstalk modulations inside the host for its survival and *pknE* contributes to these responses.

**Figure 3:** Δ*pknE* infected macrophages potentiates a crosstalk between SAPK/JNK and Erk½, and p38 and Erk½ pathways. Cells to be infected were treated with A) SAPK/JNK and B) p38 inhibitors, for 1 h and lyzed 1 h post infection. The lysates were subjected to western blotting and probed with phospho and non phospho Erk½ antibodies. The results from three independent experiments are shown. The abbreviations Ctrl denote control and LPS denotes lipopolysaccharide.

### Δ*pknE* modulates the secretion of cytokines TNF-α and IL-6 in response to intracellular signaling

The current observation on crosstalk and our previous observations [3], [15] that Δ*pknE*-infected macrophages are defective in producing pro and anti-inflammatory cytokines compelled us to assess production of TNF-α and IL-6 in the presence of pathway-specific inhibitors.

Three signaling pathways, MAPK (Erk½, p38MAPK, SAPK/JNK), survival (Akt, arginase) and apoptosis (caspase-8, caspase-9, TP53) were studied. While Erk½ inhibitor almost inhibited production of TNF-α and IL-6 in Rv-infected macrophages, increased production of these cytokines in Δ*pknE*-infected macrophages was observed as compared to Rv infected macrophages (p<0.0001, for both) (Figures 4A,4D). Δ*pknE*-infected macrophages had reduced secretion of TNF-α in the presence of p38MAPK and SAPK/JNK inhibitor (p<0.0001, p<0.001 respectively in Δ*pknE* versus Rv-infected macrophages) (Figure 4A). Secretion of IL-6 in both Rv and Δ*pknE*-infected macrophages was unaffected in the presence of p38 and SAPK/JNK inhibitors (Figure 4D).

**Figure 4:** The secretion of TNF-α and IL-6 in Δ*pknE* infected macrophages is modulated by intracellular signaling. Culture supernatants post infection in the presence of inhibitors TNF-α [A) MAPK family, B) survival family and C) caspase family] and IL-6 α [D) MAPK family, E) survival family, and F) caspase family ] was analyzed using ELISA on day 1. The error bars represent standard error of the means. Data is from three independent experiments. The symbols *, **, *** denotes p<0.05, p<0.001 and p<0.0001(one way ANOVA) respectively, when Δ*pknE* was compared to Rv infected macrophages.

In comparison with Rv-infected macrophages, Δ*pknE*-infected macrophages produced reduced amounts of TNF-α and IL-6 in the presence of Akt inhibitor (p<0.05 and p<0.0001 respectively), and arginase inhibitor had a reciprocal effect on their secretion (Figures 4B, 4E). In CΔE-infected macrophages cytokine levels were restored to that observed in Rv-infected macrophages.

Apoptosis pathway (caspase-8, 9, TP53) inhibitors did not have any effect on the secretion of TNF-α or IL-6 secretion in Rv-infected macrophages (Figures 4C, 4F). However, in Δ*pknE*-infected macrophages secretion of TNF-α was decreased in the presence of caspase-8 inhibitor as compared to Rv infected macrophages (p<0.05). IL-6 was modestly increased in Δ*pknE*-infected macrophages in the presence of caspase-8/9 and TP53 inhibitors, of which only caspase-9 inhibition was significant (p<0.05) (Figure 4F). CΔE-infected macrophages had cytokine levels comparable to that of Rv-infected macrophages. Collectively, these data show that secretion of TNF-α and IL-6 is influenced by the genes of MTB that enable crosstalk between intracellular pathways in the host and that *pknE* plays a significant role in crosstalk response thereby modulating the secretion of inflammatory cytokines.

### Nitrate stress response

From our previous observations [3], [15] we found that *pknE* has a role in nitrate stress response suppressing the host cell apoptosis. The role of *pknE* in modulating intracellular signaling in response to nitrate stress was studied using an exogenous NO donor, sodium nitroprusside.

Phosphorylation of p38MAPK was higher in Δ*pknE*-infected macrophages while Erk½ and SAPK/JNK were reduced in Δ*pknE*-infected macrophages, similar to that observed in the absence of NO donor (Figures 5A, 5B and 5C). Phosphorylation of ATF-2 was increased in Δ*pknE*-infected as compared to Rv-infected cells (p<0.05, Figure 5D), but phosphorylation of c-JUN was similar in both Rv and Δ*pknE*-infected macrophages (data not shown). Phosphorylation of NF-kB was reduced in Δ*pknE*-infected as compared to Rv-infected macrophages (p<0.05) (Figure 5E). CΔE-infected macrophages had the restored phenotype of Rv-infected macrophages. Thus, in the presence of NO stress Δ*pknE*-infected macrophages reproduced events observed in the endogenous NO host response. This clearly proves that *pknE* responds to NO stress in the host and by modulating signaling events enables the intracellular survival of MTB.

**Figure 5:** Δ*pknE* infected macrophages show defective MAPK signaling in the presence of NO stress. Controls (ctrl, LPS) and infected cells were lysed post NO stress and subjected to western blotting. The blots were probed with phospho A) Erk1/2, B) p38, and C) SAPK/JNK with their respective non phospho antibodies and the results of three independent experiments are given. The corresponding densitometry values of phospho and nonphospho are given at the end of antibody probed blots. *** denotes p<0.0001, when Δ*pknE* infected macrophages compared with Rv (one – way ANOVA). The abbreviations ctrl denotes control, LPS denotes lipopolysaccharide, and NO denotes nitric oxide. Nuclear fractions isolated post infection was subjected to DNA binding ELISA D) ATF-2 and E) NF-kB. The results are from three independent experiments. The error bars denote standard error of the means. * denotes p<0.05 (one way ANOVA) when Δ*pknE*+NO was compared to Rv+NO treated macrophages.

### Δ*pknE*-infected macrophages modulate the expression of receptors for HIV entry

The role of *pknE* in the modulation of CCR5 and CXCR4 receptors involved in HIV entry was investigated based on our observation that Δ*pknE* has defective MAPK signaling, and the knowledge that MAPK signaling influences modulation of coreceptors.

The expression kinetics of CCR5 and CXCR4 was examined on days 1 and 2 post-infection. Expression of CCR5 was reduced in Δ*pknE*-infected macrophages as compared to Rv-infected macrophages on both days (p<0.05; Figure 6A). Conversely, expression of CXCR4 was increased in macrophages infected with Δ*pknE* when compared to Rv-infected macrophages (p<0.05; Figure 6E). CΔE-infected macrophages had comparable levels of coreceptor expression to that of Rv-infected macrophages.

**Figure 6:** Δ*pknE* infected macrophages modulate the expression of coreceptors CCR5 and CXCR4 by intracellular cascades. Cells post infection were stained with CCR5 (A) and CXCR4 (E) antibody and the expression was analyzed in a time dependent manner using FACS, * denotes p<0.05 (Twoway – Anova) when Δ*pknE* was compared to Rv infected macrophages. Cells post infection in the presence of inhibitors CCR5 [B) MAPK family, C) survival family and D) TP53] and CXCR4 [F) MAPK family, G) survival family, and H) caspase family] expression was analyzed on day1 post infection using FACS. The symbols *, **, ***denotes p<0.05, p<0.001 and p<0.0001 respectively (one way – Anova) when Δ*pknE* was compared to Rv infected macrophages.

### Reduction in CCR5 by Δ*pknE*-infected macrophages is influenced by intracellular signaling cascades

Our previous [15] and present findings, persuaded us to examine the modulation of HIV receptors by MAPK, survival and apoptosis family of inhibitors. While MAPK inhibitors reduced the expression of CCR5 in Δ*pknE*-infected macrophages (p<0.05), SAPK/JNK inhibitors increased the expression of CCR5 in comparison with Rv-infected cells (Figure 6B). Akt inhibition did not have any effect on CCR5 expression (Figure 6C). Δ*pknE*-infected macrophages had increased expression of CCR5 in the presence of arginase inhibitor as compared to Rv-infected macrophages (p<0.001; Figure 6C). In the presence of TP53 inhibitor, both Rv and Δ*pknE*-infected macrophages had greater reduction in the expression of CCR5 (Figure 6D). CΔE-infected macrophages were able to restore the expression levels similar to Rv-infected macrophages.

### Increase in CXCR4 by Δ*pknE*-infected macrophages is influenced by intracellular signaling cascades

Modulation of CXCR4 expression was also assessed in the presence of MAPK, survival and apoptosis inhibitors. In general, MAPK and Akt inhibitors increased the expression of CXCR4 in Rv-infected macrophages. In contrast, Δ*pknE*-infected macrophages had significantly reduced CXCR4 expression in the presence of Erk½ inhibitor (p<0.0001, Figure 6F) and moderate reduction in the presence of p38MAPK and SAPK/JNK inhibitors, compared to Rv infected macrophages (Figure 6F). Akt inhibitor did not affect expression of CXCR4 (Figure 6G), but arginase inhibitor reduced the expression of CXCR4 in Δ*pknE*-infected macrophages (p<0.05 when compared to Rv-infected cells) (Figure 6G). TP53 inhibitor reduced the expression of CXCR4 in Rv, Δ*pknE* and CΔE-infected macrophages (Figure 6H). CΔE-infected macrophages reversed the changes observed in Δ*pknE*-infected macrophages.

### Δ*pknE* modulates coinfection of MTB-infected THP-1 cells and MDM with HIV

THP-1 macrophages and MDM were coinfected with an MTB strain (Rv, Δ*pknE* and CΔE) and a CCR5 (R5) or CXCR4 (X4)-tropic HIV strain to examine the effect of coreceptor modulation on HIV entry and infection, by measuring HIV-1 p24 antigen levels in infected culture supernatants. While THP-1 macrophages coinfected with Δ*pknE* and R5-tropic virus had reduced p24 levels, cells coinfected with X4 virus had increased p24 levels (See Table S1). This validates our finding that Δ*pknE*-infected macrophages had increased CXCR4 and decreased CCR5 expression.

To further confirm these findings, coinfection was performed in MDM obtained from normal healthy individuals. In MDM model of infection, p24 antigen levels were increased in Δ*pknE*-infected macrophages coinfected with R5 as well as X4-tropic viruses as compared to Rv-coinfected cells (p<0.05, Figures 7A,7C). Further, in the presence of SAPK/JNK inhibitor, Δ*pknE*-infected macrophages coinfected with R5 as well as X4-tropic viruses had higher p24 antigen levels as compared to Rv-coinfected macrophages (p<0.05, Figures 7B,7D).

**Figure 7:** Δ*pknE* coinfected with CCR5 and CXCR4 tropic HIV-1 increases p24 levels in MDMs. Human monocyte derived macrophages (n = 6), were infected with *M. tuberculosis* strains followed by coinfection with a CCR5 tropic virus in the presence (A), and absence of SAPK/JNK inhibitor (B). Similarly, coinfection was performed using CXCR4 tropic virus in the presence (C) and absence of SAPK/JNK inhibitor (D). p24 antigen levels were estimated using ELISA on day 4. * denotes p<0.05 (one way – Anova) when Δ*pknE* was compared to Rv infected macrophages.

The observations of increased p24 levels in macrophages coinfected with R5 tropic virus and Δ*pknE* corroborates increased CCR5 expression observed in Δ*pknE* infected macrophages treated with SAPK/JNK inhibitor. Further, decreased p24 levels in R5 tropic virus and Rv coinfected macrophages confirms decreased CCR5 expression observed in RV infected macrophages treated with SAPK/JNK inhibitor. This data for the first time shows that *pknE* contributes to the co-pathogenesis of HIV by modulating intracellular signaling in the host.

## Discussion

Virulence and infectivity of MTB modulates various apoptotic paradigms thereby reducing immunity of the host [18], [19]. *pknE* of MTB suppresses cell death of the host by inhibiting intrinsic pathway of apoptosis and arginase2 dependent mechanisms [15]. MAPK signaling in eukaryotes plays an important role in cytokine and apoptosis regulation [10], [20]. The present study investigates the role of *pknE* in modulating MAPK cascades and its impact on HIV/TB coinfection.

Analysis of MAPK signaling showed Δ*pknE*-infected macrophages to have decreased Erk½ phosphorylation. This observation corresponds with our previous finding that Δ*pknE*-infected macrophages had reduced phosphorylation of Akt, an upstream activator of Erk½ [15], correlating the findings of Yang et al [21]. In addition, selective inhibition of p46SAPK/JNK was observed in Δ*pknE* infected macrophages. These inferences prompted us to examine the phosphorylation kinetics of transcription factors c-JUN, ATF-2 and NF-kB that are regulated by MAPK cascades. Phosphorylation of c-JUN and ATF-2 were dramatically delayed and reduced in Δ*pknE* as compared to Rv-infected macrophages.

This defective MAPK signaling could be a reason for the Δ*pknE* infected macrophages to have dampened cytokine secretion and execute apoptosis independent of extrinsic pathway (TNF-α) and iNOS [15]. This concurs with previous findings that c-JUN and ATF-2 induces the secretion of TNF-α, activating p46SAPK/JNK and iNOS [22], [23]. The current data suggest that deletion of *pknE* results in deactivation of survival pathways inside the host. This underlines the role for *pknE* in modulating host intracellular cascades.

Use of pathway specific inhibitors to confirm the defective MAPK signaling in Δ*pknE*-infected macrophages did not reverse the effects. However, the secretion of TNF-α and IL-6 were modulated by inhibitors to various intracellular pathways. Observations from the inhibitor studies suggested the probability of crosstalk responses and Δ*pknE* infected macrophages had cross talk responses between Erk½ and SAPK/JNK, and p38MAPK and Erk½ pathways. This is in concordance with earlier studies where crosstalks within MAPK signaling were reported [17]. Our study for the first time demonstrates the role of *pknE* in crosstalk responses essential for the intracellular survival of MTB.

In our earlier observations *pknE* was found to respond NO stress that results in suppression of apoptosis [3], [15]. In the present study, the function of *pknE* in modulating intracellular signaling in response to the NO stress of the host was examined using SNP as NO donor that mimics *in vivo* situations of NO stress [24]. As expected, Δ*pknE*-infected macrophages had reduced phosphorylation of MAPKs that confirms *pknE* in modulating intracellular signaling during NO stress of the host.

Our findings suggest that *pknE* increases Erk½ signaling thereby suppressing apoptosis which favors the survival of MTB. This is analogous with a previous report where Erk½ was shown to suppress apoptotic signals [25].

In the next part of the study we endeavored to analyze the significance of *pknE* in the co-pathogenesis of HIV. This was investigated since the data about mycobacterial genes involved in HIV coinfection remains unexplored. Nevertheless earlier reports have shown MAPKs, Akt, chemokines, apoptosis, IL-12 and MTB to modulate CCR5 and CXCR4 coreceptors involved in HIV entry [26]–[32].

Here we found that THP-1 macrophages infected with Δ*pknE* suppressed CCR5 but increased CXCR4 expression as compared to the wild-type strain. This finding was further confirmed by coinfection studies with MTB and HIV-1 tropic strains. Next we examined various intracellular pathways that could influence this modulation. MAPK and arginase signaling were found to play an important role in the expression of CCR5 and CXCR4 in macrophages infected with Δ*pknE*.

For the first time, we show that Δ*pknE* induces apoptosis and down modulates intracellular events that suppress CCR5 expression. This concurs with a previous study where CCR5 was shown to induce antiapoptotic signals via Akt and Erk½ [32]. The modulations of coreceptor expression were further investigated in MDM derived from normal healthy individuals. In contrast to THP-1 model of coinfection, Δ*pknE* increased the levels of p24 antigen upon coinfection with either R5 or X4 tropic HIV-1 strains. Among the MAPK and arginase signaling, SAPK/JNK was chosen for further validation. Inhibition of the SAPK/JNK signaling and coinfection with either R5 or X4 tropic HIV-1 strains increased the p24 antigen levels in Δ*pknE* coinfected macrophages. However inhibition of SAPK/JNK signaling markedly reduced the p24 levels in macrophages coinfected with either R5 or X4 tropic HIV-1 strains and Rv. These data suggests SAPK/JNK signaling as one among the cascade that regulates CCR5/CXCR4 expression. This is in concordance with an earlier report where inhibition of SAPK/JNK was shown to reduce CCR5 expression [28].The reasons for disparity in coinfection studies between THP-1 and MDM cells could be multifactorial including differences in CD4 receptor expression, genetic composition of the host, etc [33]. In contrast to our study, p38 signaling was reported to regulate the expression of coreceptors upon infection with MTB [34]. Our study using various pathway specific inhibitors and HIV/TB model of coinfection authenticate the significance of SAPK/JNK pathway in regulating the coreceptor expression.

In conclusion, our previous [3], [15] and the current findings show that *pknE* contributes to the intracellular survival of MTB by initiating crosstalks within the intracellular signaling of the host. This protective strategy employed by MTB provides a favorable niche for HIV infection.

## Supporting Information

Table S1 **Δ** ***pknE*** **coinfected with CCR5 has reduced while with CXCR4 have increased p24 levels in THP-1 model of coinfection.** THP-1 derived macrophages were infected with *M. tuberculosis* strains followed by coinfection with a CCR5 and CXCR4 tropic virus. The p24 antigen levels were estimated using ELISA on day 4. *, ** denotes p<0.05 and p<0.001 (one way – Anova) when Δ*pknE* was compared to Rv infected macrophages.
(DOC)
